The article "Utility of Optical Coherence Tomography Angiography (OCTA) in Granulomatosis With Polyangiitis" was published in 2022. Journal: Cureus.

# Utility of Optical Coherence Tomography Angiography (OCTA) in Granulomatosis With Polyangiitis

**DOI:** 10.7759/cureus.22612

**Published:** 2022-02-25

**Authors:** Salil Mehta, Neena Chitnis, Amey Medhekar

**Affiliations:** 1 Department of Ophthalmology, Lilavati Hospital and Research Center, Mumbai, IND; 2 Department of Rheumatology, Lilavati Hospital and Research Center, Mumbai, IND; 3 Department of Internal Medicine, Lilavati Hospital and Research Center, Mumbai, IND

**Keywords:** immunosuppressive treatment, anterior ischemic optic neuropathy, retinal vasculitis, wegener's granulomatosis, optical coherence angiography

## Abstract

A 61-year-old male presented with visual loss in the left eye. A CT scan of the chest revealed multiple lung cavities in both lungs. He had a positive C-ANCA suggestive of granulomatosis with polyangiitis. There were multiple areas of superficial retinal opacification in the right eye and anterior ischemic optic neuropathy in the left eye. An optical coherence tomography (OCT)/optical coherence tomography angiography (OCTA) revealed areas of superficial capillary dropout and areas of flow void in the choriocapillaris. The patient underwent immunosuppressive therapy and at follow-up, there was a reduction in the flow voids. Use of the OCT/OCTA allowed us to detect clinically visible and occult retinal/choroidal ischemia/inflammation and monitor response.

## Introduction

Systemic vasculitis, such as granulomatosis with polyangiitis or polyarteritis nodosa, are common immune-mediated diseases with a myriad of systemic and ocular findings. Diagnosis is often complex or delayed. Ocular manifestations include scleritis, keratitis, cotton wool spots, and choroidal lesions. We report the ocular and systemic findings of a patient with granulomatosis with polyangiitis who manifested retinal and choroidal lesions and systemic granulomatous disease. The patient underwent a complete ophthalmic evaluation and detailed optical coherence tomography/optical coherence tomography angiography (OCT/OCTA) studies using a Topcon DRI OCT Triton Plus swept-source OCT system (Topcon Healthcare, Oakland, NJ). OCTA permits in vivo retinal vasculature assessment of both the superficial and deep retinal plexus as well as the choroid [1]. Importantly, this test does not use intravenous sodium fluorescein, thus eliminating all risks of anaphylaxis. We were able to detect retinal and choroidal inflammation that resolved following immunosuppressive treatment.

## Case presentation

A 61-year-old gentleman, a known pre-diabetic, presented with complaints of profound visual loss in the left eye, along with tiredness, weakness, significant weight loss (10 kgs), and dry cough since the last three months. On admission, he was afebrile, with a pulse rate of 92/min and a blood pressure reading of 120/70 mmHg. Clinical examination of the cardiovascular and respiratory systems was non-contributory. 

The article "Utility of Optical Coherence Tomography Angiography (OCTA) in Granulomatosis With Polyangiitis" was published in 2022. Journal: Cureus.

Relevant investigations revealed anemia (hemoglobin: 10 gm/dl; normal 13-17 gm/dl) with neutrophilic leukocytosis (total leucocyte count: 19.04 thousands/mm3; normal 4-10 thousands/mm3 with absolute neutrophil count 17.10 thousands/mm3; normal 2-7 thousands/mm3). Erythrocyte sedimentation rate (ESR) was elevated at 89 mm/hr (normal 0-10mm/hr) as was the C-reactive protein (CRP) at 266.62 mg/l (normal <5.0 mg/l). His renal function as assessed by serum creatinine measurements was normal at 1.04 mg/dl (normal 0.70 - 1.20 mg/dl), confirming the absence of pauci-immune glomerulonephritis, an antibody associated vasculitis (AAV) phenomenon. His prediabetic status was suggested by his glycosylated hemoglobin value of 6.4% (normal: 4-5.6%; pre-diabetic state 5.7-6.4%) with a fasting blood sugar level of 136 mg/dl (normal < 130 mg/dl). Serum electrophoresis revealed a diffuse increase in the gamma globulin region (2.11 gm%; normal 0.7-1.7 gm%).

A CT scan of the chest revealed multiple varying-sized, cavitary nodular lesions in both lung fields, the largest measuring 3.5 X 3 cm in the right upper lobe, along with few centrilobular nodular opacities in the right middle lobe (Figure 1).

**Figure 1:** Coronal CT scan of the chest showing a large cavitary lesion in the right lung (marked by an arrow)

These findings were suggestive of a fungal infection or granulomatosis. A scan of the abdomen and pelvis revealed multiple hypoenhancing lesions in the splenic parenchyma suggestive of infarcts. A CT-guided core biopsy from the lung revealed large areas of caseation necrosis and multiple granulomas composed of epithelioid cells suggestive of granulomatous inflammation. Ziehl-Neelsen (ZN) staining for acid-fast bacilli and periodic acid Schiff (PAS) stains for fungi were negative. A GeneXpert test for mycobacterium was negative.

An auto-antibody profile revealed negative results for ANA (anti-nuclear antibody; by quantitative immunofluorescence method); anti-DS-DNA (anti-double-stranded DNA; by serum enzyme immunoassay) and p-ANCA (anti-MPO; perinuclear antineutrophil cytoplasmic antibodies). C-ANCA (anti-PR3; by serum enzyme immunoassay) was strongly positive at 288.9 RU/ml (positive > 20 RU/ml), suggestive of granulomatosis with polyangiitis (GPA).

On examination, visual acuity was 6/6 in the right eye and hand motions close to the face in the left eye. Examination of the anterior segments bilaterally was normal except for a left relative afferent pupillary defect. Fundus examination revealed a clear vitreous with multiple areas of superficial retinal opacification within the macula of the right eye. The size and appearance of these areas were inconsistent with standard descriptions of cotton wool spots (Figure 2).

The article "Utility of Optical Coherence Tomography Angiography (OCTA) in Granulomatosis With Polyangiitis" was published in 2022. Journal: Cureus.

**Figure 2:** Fundus photo of the right eye with areas of retinal opacification, as shown by the arrows

The left eye revealed a pale edematous optic disc with peripapillary hemorrhages consistent with anterior ischemic optic neuropathy (Figure 3).

**Figure 3:** Fundus photo of the left eye showing a pale edematous optic disc (anterior ischemic optic neuropathy, AION) (a large arrow marks the optic nerve head)

OCT/OCTA of the right eye revealed areas of capillary dropout in the superficial capillary plexus, consistent with the areas of retinal opacification and suggestive of vasculitis (Figure 4).

**Figure 4:** Pre-treatment OCTA of the superficial capillary plexus with an area of capillary drop-out corresponding to the retinal opacification (marked by a white arrow) OCTA: optical coherence tomography angiography

The choriocapillaris demonstrated multiple discrete areas of flow void consistent with choriocapillaris inflammation (Figure 5).

**Figure 5:** Pre-treatment OCTA showing multiple areas of flow void in the choriocapillaris (representative areas marked by arrows) OCTA: optical coherence tomography angiography

A B-scan through the area of opacification showed uniform hyperreflectivity across the internal retinal layers (Figure 6).

**Figure 6:** Structural OCT B-scan passing through an area of flow void demonstrating uniform hyperreflectivity throughout the inner retina, as marked by the vertical arrow. OCT: optical coherence tomography

Similar studies could not be performed in the left eye due to poor fixation.

The patient underwent intensive immunosuppressive therapy with intravenous methylprednisolone (500 mg) for three days, followed by a single cycle of intravenous cyclophosphamide (500 mg), and was discharged on oral prednisolone (50 mg/daily, tapering by 10 mg every 10 days).

At the one-month follow-up, the visual acuities were unchanged. Fundus exam revealed a significant reduction of retinal opacification in the right eye while optic atrophy was seen in the left eye. An OCTA revealed a marked reduction in the superficial capillary dropout as well as the choriocapillaris flow voids of the right eye (Figure 7).

**Figure 7:** Post-treatment OCTA showing reduction of flow void areas in the choriocapillaris OCTA: optical coherence tomography angiography

## Discussion

Granulomatosis with polyangiitis is a granulomatous vasculitis that involves small and medium-sized vessels, and ocular findings may eventually occur in up to 28-87% of patients. Ocular anterior segment findings include episcleritis, scleritis, and peripheral ulcerative keratitis. The orbit is often involved usually due to disease in the paranasal sinuses and may present as proptosis. Retinal or choroidal involvement is seen in 5-12% of patients and lesions include cotton wool spots, hemorrhages, vascular occlusions, or choriocapillaritis [2].

The article "Utility of Optical Coherence Tomography Angiography (OCTA) in Granulomatosis With Polyangiitis" was published in 2022. Journal: Cureus.

Pathological studies of the choroid have revealed multiple foci of granulomatous inflammation largely by epithelioid cells with lymphocytes and scattered multinucleated giant cells. In several areas, the choriocapillaris is infiltrated by inflammatory cells and the capillaries are blocked by inflammatory debris. Occasional foci of fibrinoid necrosis are seen in the choroid in proximity to the choriocapillaris [3].

Mirza et al. described the findings of a 58-year-old male with proven granulomatosis with polyangiitis. The left eye showed findings of central retinal arterial occlusion and in the right eye, the posterior pole revealed discrete choroidal lesions. Fundus fluorescein angiography (FFA) showed early blocked choroidal fluorescence with little evidence of filling in the later phase suggestive of bilateral choroidal infarcts [4].

Iida and co-workers have described a 64-year-old male with central retinal arterial occlusion in one eye and branch retinal arterial occlusion in the other eye. Indocyanine green angiography (ICG) showed a widespread filling defect of choroidal arteries and the choriocapillaris bilaterally. The authors postulated that the chorioretinal ischemia may have been due to vasculitis, leading to occlusion of retinal circulation or the short posterior ciliary arteries [5].

The patient we describe had retinal ischemia in the right eye and anterior ischemic optic neuropathy in the left eye. The OCTA revealed areas of capillary dropout in the superficial capillary plexus with extensive areas of flow void within the choriocapillaris. Following a single pulse treatment of cyclophosphamide, there was a significant reduction in both the size of superficial capillary plexus dropout as well as the areas of choriocapillaris flow void. Additionally, the use of OCT/OCTA allowed us to detect occult choroidal lesions not visible on clinical examination. Previous case reports have documented choroidal ischemia via ICG or FFA [4-5]. FFA remains the gold standard for the diagnosis of posterior segment inflammation but the high-resolution imagery of OCT/OCTA permitted adequate visualization of lesions in this patient.

A potential differential diagnosis for the choriocapillaris flow voids is the presence of choroidal granulomas as occur in tuberculosis or sarcoidosis. These granulomas are commonly well-visualized, round in shape, with well-demarcated margins, are hyporeflective vis-a-vis the rest of the choroid, and are best seen on enhanced depth imaging (EDI) studies [6]. The sectional B-scan we describe does not show any obvious granulomas.

The article "Utility of Optical Coherence Tomography Angiography (OCTA) in Granulomatosis With Polyangiitis" was published in 2022. Journal: Cureus.

We feel that the superficial capillary dropout as well the choriocapillaris flow voids we describe are OCT/OCTA manifestations of inflammation within the retinal and choriocapillaris layers due to their marked improvement following corticosteroid treatment and the absence of other structural lesions such as granulomas.

Several cases of optic neuropathy have been described as either compressive lesions as part of granulomatous inflammation of the orbit [7] or isolated vasculitic processes involving the optic nerve [8-9]. Quist et al. describe the case of a previously healthy 50-year-old woman with anterior ischemic optic neuropathy due to granulomatosis with polyangiitis. The authors note standard protocols that mandate diagnostic tests for temporal arteritis such as a suggestive history (jaw claudication, scalp tenderness, or palpable temporal artery), ESR, or temporal artery biopsies but point out that other forms of vasculitis are likely and should be kept in mind [8]. Similarly, in our case, the ANCA-associated vasculitis was the likely pathogenic mechanism for the optic neuropathy and temporal arteritis was considered unlikely due to the absence of suggestive history.

We performed a literature search on PubMed with the keywords granulomatosis with polyangiitis AND OCT/OCT angiography and were able to retrieve one previous report that discusses the potential role of OCT/OCTA in the management of granulomatosis with polyangiitis. Takashi et al. described a 36-year-old male with the fundus findings of a retinal pigment epithelial (RPE) detachment and a serous retinal detachment (SRD). They used OCTA to evaluate blood flow within the structure of the SRD to rule out an underlying choroidal neovascular membrane [10].

## Conclusions

We describe the systemic and ocular findings of a case of granulomatosis with polyangiitis with widespread disease. This included lung, gastrointestinal, and ocular sites of inflammation. The use of OCT/OCTA allowed us to characterize the retinal and choroidal lesions as consistent with retinal vasculitis and choriocapillaritis. The choroidal disease was more extensive than the clinical examination would suggest. We could also monitor its response to immunosuppressive therapy, thus suggesting a potential role for this modality in short and long-term follow-ups.

The article "Utility of Optical Coherence Tomography Angiography (OCTA) in Granulomatosis With Polyangiitis" was published in 2022. Journal: Cureus.

The ease of use, high-resolution imagery, and safety profile, especially for repeated follow-ups, suggest an increasing role for OCT/OCTA in patients with systemic vasculitis that involves the retinal-choroidal region.
